RETRACTED

# Occurrence of L1014F and L1014S mutations in insecticide resistant *Culex quinquefasciatus* from filariasis endemic districts of West Bengal, India

**DOI:** 10.1371/journal.pntd.0010000

**Published:** 2022-01-13

**Authors:** Priyanka Rai, Dhiraj Saha

**Affiliations:** Insect Biochemistry and Molecular Biology Laboratory, Department of Zoology, University of North Bengal, P.O. North Bengal University, Siliguri, District - Darjeeling, West Bengal, India; Kenya Agricultural and Livestock Research Organization, KENYA

## Abstract

**Introduction:**

Lymphatic filariasis causes long term morbidity and hampers the socio-economic status. Apart from the available treatments and medication, control of vector population *Culex quinquefasciatus* Say through the use of chemical insecticides is a widely applied strategy. However, the unrestrained application of these insecticides over many decades has led to resistance development in the vectors.

**Methods:**

In order to determine the insecticide susceptibility/resistance status of *Cx*. *quinquefasciatus* from two filariasis endemic districts of West Bengal, India, wild mosquito populations were collected and assayed against six different insecticides and presence of L1014F; L1014S kdr mutations in the voltage-gated sodium channel gene was also screened along with the use of synergists to evaluate the role of major detoxifying enzymes in resistance development.

**Results:**

The collected mosquito populations showed severe resistance to insecticides and the two synergists used–PBO (piperonyl butoxide) and TPP (triphenyl phosphate), were unable to restore the susceptibility status of the vector thereupon pointing towards a minor role of metabolic enzymes. kdr mutations were present in the studied populations in varying percent with higher L1014F frequency indicating its association with the observed resistance to pyrethroids and DDT. This study reports L1014S mutation in *Cx*. *quinquefasciatus* for the first time.

## Author summary

Lymphatic filariasis is caused by a nematode worm *Wuchereria bancrofti* and transmitted by mosquito vector *Culex quinquefasciatus*. The vector *Culex quinquefasciatus* is a nuisance due to its biting habit and involvement in transmission of many deadly diseases in the tropics and sub tropics. Therefore, to control disease transmission by mosquito vectors, humans have been relying on the use of chemical insecticides since many decades. However, the over and unplanned application of insecticides has led to insecticide resistance in the mosquito population. As such, the insecticides have failed to produce 100 percent mortality in the mosquito vectors. This scenario is an important and urgent issue of concern because apart from medical treatment, major reliance for the control of vector-borne diseases still lies on the use of chemical insecticides targeted against the mosquito vectors. Moreover, there is a need to survey and evaluate insecticide susceptibility/resistance status of mosquito vectors along with the underlying mechanisms of resistance in national and regional level to draw an idea about the existing insecticide resistance pattern. This will further help in designing efficient vector control strategies in the near future on both national and regional basis.

RETRACTED

## 1. Introduction

*Culex quinquefasciatus* commonly known as the southern house mosquito is widely distributed in tropical and subtropical regions. *Culex quinquefasciatus* is the most abundant species of mosquito in the sub-Himalayan region of West Bengal [1,2]. This mosquito species is opportunistic and may breed and habituate any temporary collection of stagnant water apart from its other natural breeding habitat- drains, stagnant puddles of water, cemented channels, muddy pools and water-filled artificial containers. *Culex quinquefasciatus* serves as a vector for many diseases like lymphatic filariasis, West Nile Fever, Saint Louis Encephalitis [3] and even act as a bridge to transport slyvatic arboviruses from bird to mammals [4,5]. Some studies suggest its role in transmission of Zika virus [6] and *Plasmodium relictum* that cause avian malaria [7]. In Southeast Asia, *Cx*. *quinquefasciatus* is a primary vector of lymphatic filariasis which is one of the most important Neglected Tropical Diseases (NTDs) and ranks second in causing long term morbidity in the human society [8]. Negative impact of the disease on the socio-economic status of an individual is also non-negligible.

Although there are drugs and treatments available to combat lymphatic filariasis and the disease was aimed to be eradicated by the year 2020 [8], management of vector population through the use of chemical insecticides is still one of the major strategies of disease control. In India, 257 districts in 21 states and Union territories are endemic to filariasis with a probability of affecting approximately 650 million population [9]. Ministry of Health and Family Welfare, Government of India, have designed ‘Twin pillar strategies’ that include Mass Drug Administration (MDA) for prevention of disease transmission and Morbidity Management and Disability Prevention (MMDP) for taking care of infected patients for elimination of filariasis in India. In the state West Bengal, 12 districts are reported to be endemic to the disease where Coochbehar and Malda are the only two districts of northern West Bengal that are endemic to lymphatic filariasis [9]. Apart from disease control programmes and strategies like mass drug administration (MDA), proper sanitation and hygiene to check the spread of disease, vector control and management also form an important aspect regarding the control of the proliferation of mosquito-borne diseases in these two districts. Synthetic insecticides in the form of indoor residue spraying, insecticide impregnated bed nets and outdoor fogging is in use since many decades to control vector-borne diseases and nuisance caused by mosquitoes. WHO has approved the use of 4 classes of insecticides *i*.*e*., pyrethroids, organophosphates, organochlorines and carbamates to be applied against mosquito vectors [10]. However, the continuous exploitation of these insecticides on the mosquito vectors led to the development of insecticide resistance.

RETRACTED

Of the four mechanisms of insecticide resistance development in mosquitoes, metabolic detoxifying enzymes and target-site insensitivity have been widely studied and known as the prime mechanism of resistance in the vector population [10]. Resistance involving the major detoxifying enzymes occurs either by an enhanced enzyme action or by a qualitative increase in the number of isozymes [11,12]. Target-site insensitivity on the other hand occurs as a result of mutation in the target receptor at the neurological site of an insect to which a particular insecticide binds [13]. Carbamate and organophosphate insecticides target the acetylcholinesterase enzyme (AChE) [14], while the other two groups- synthetic pyrethroids and DDT attack the voltage-gated sodium channel in the neuron membrane which results in prolonged opening of the channel causing involuntary muscle spasms and death, a condition termed as the knock down effect [14,15]. With the rising problem of DDT resistance in mosquito vectors, in the mid-1970s synthetic pyrethroids in the form of deltamethrin, cypermethrin and permethrin were introduced for mosquito vector control. However, excessive use of DDT in the past and synthetic pyrethroids in present to combat the agricultural pests and vectors carrying many human diseases have resulted in the development of resistance in the pest population known as knock down resistance (kdr) through point mutation in the sodium channel gene, thereby rendering the channel unfit for insecticide binding. Mutation in the 1014 position of voltage-gated sodium channel gene from Leucine to Phenylalanine (L1014F) is the most common kdr mutation found in *Culex sp*. and the only kdr mutation found in *Cx*. *quinquefasciatus*. In *Culex sp*., the L1014S mutation (Leucine to Serine) has only been found in *Cx*. *pallens* and *Cx*. *pipiens* until now.

RETRACTED

The objective of this study was to map resistance status of *Cx*. *quinquefasciatus* from two lymphatic filariasis endemic districts of West Bengal against different insecticides and to screen the presence of kdr mutations in the sodium channel gene associated with insecticide resistance. The involvement of metabolic enzymes in resistance development through synergistic assays was also evaluated.

## 2. Material and methods

### 2.1. Ethics statement

The Institutional Animal Ethics Committee (IAEC) Department of Zoology, University of North Bengal (Regn no. 840/GO/Re/S/04/CPCSEA) granted a waiver for ethics approval as there was no human trail or higher vertebrates involved in the present study. The IAEC also approved the use of rat for blood feeding (approval no. IAEC/NBU/2019/19). All procedures were performed in accordance with relevant guidelines of the IAEC and ARRIVE.

### 2.2. Study area

Field *Cx*. *quinquefasciatus* populations for the study were collected from two districts of West Bengal, India- Coochbehar and Malda (Fig 1). These two districts out of total eight districts in northern West Bengal are endemic to the disease lymphatic filariasis. These districts have a tropical climate with four seasons–dry season (March–April), rainy season (May–September), autumn season (October) and winter season (November–February). The northern part of West Bengal receives an annual rainfall of 200–400 cm and has an average temperature range of about 30°C during summers. Coochbehar district has a population of about 2.82 million and Malda about 3.9 million, both share international borders with Bangladesh [16]. Therefore, insecticide susceptibility mapping of wild *Cx*. *quinquefasciatus* was carried in these two districts owing to their disease endemicity, dense population, poor sanitation and infrastructure.

**Fig 1:** Map showing six sampling sites in two districts of northern part of West Bengal. (Figure created using QGIS software version 3.22. Shape file of India and West Bengal downloaded from: https://www.naturalearthdata.com/downloads/10m-cultural-vectors/).

### 2.3. Mosquito collection

Mosquito larvae and pupae were collected from 3 densely populated sites in Coochbehar and Malda districts (Table 1 and Fig 1) and was labeled as F0. Sampling was conducted from January 2019—February 2020 from natural breeding habitats of *Culex sp–*drains, stagnant water, pools, plastic containers, sewers and cemented channels. A 500 ml plastic beaker was used for the purpose and 8–10 dips were made at a particular sampling site. Average larval density was calculated for each sampling site. Prior permission from land owners were taken when sampling from private areas and from Officer-in-charge for sampling from Government areas. In the laboratory, *Cx*. *quinqueasciatus* larvae and pupae were identified following standard mosquito identification keys [17] and reared to F1 generation under controlled laboratory conditions. Adult bioassay test and kdr mutation screening was performed with the F1 generation in order to maintain population homogeneity.

RETRACTED

**Table 1:** Sampling details of *Cx*. *quinquefasciatus* from Coochbehar and Malda districts of West Bengal.

Sampling site	Coordinates	District	Nature of habitat	Total mosquito collected	Average larval density /500 ml	Co-existence of other species
Coochbehar Town (COB)	26.3452°N, 89.4482°E	Coochbehar	Muddy drains, stagnant water body	2,654	798.20	*Anopheles sp*., chironomids
Tufanganj (TFG)	26.3305°N, 89.6675°E		Cemented drains, channels	2,820	841.40	Chironomids, drain flies
Mekhliganj (MEK)	26.3474°N, 88.9102°E		Muddy pool of water, channels	3,281	822.10	Drain flies
Malda town (MLT),	25.0166°N, 88.1305°E	Malda	Stagnant puddles, cemented drains	3,590	813.30	*Anopheles sp*., drain flies
Samsi (SAM)	25.2735°N, 88.0040°E		Cemented channels, muddy drains	2,796	769.50	Chironomids, drain flies
Harichchandrapur (HCP)	25.4068°N, 87.8669°E		Muddy drains, muddy pool	2,200	489.20	Drain flies

### 2.4. Laboratory rearing of susceptible mosquito population

Susceptible population of *Cx*. *quinquefasciatus* was reared in laboratory following the protocol [18]. Larvae and pupae of *Cx*. *quinquefasciatus* were collected from drains and stagnant puddles in and around the medicinal garden of University of North Bengal (26.71°N, 88.35°E) located at a rural area of Darjeeling District. The University medicinal garden is organically maintained therefore, mosquito larvae collected were earlier not exposed to insecticides. The sample was brought to the laboratory and kept in enamel trays. Pupae were separated in 1000 ml glass beakers to avoid over-crowding and covered with a mosquito net. Larvae were provided with ground fish feed (Optimum mini pellets; made in Thailand) and newly emerged adults with cotton balls soaked in 5% sucrose solution (Merck cat. no. 61806905001730), as food source. Three to four days old female mosquitoes blood fed on trimmed rat kept in a cage inside the rearing setup. Tap water boiled with hay and then cooled to room temperature was placed in a glass beaker and served as the egg laying apparatus. Egg rafts were transferred to another enamel tray where the eggs hatched into first instar larvae. During the entire rearing period, a temperature of 25 ± 2°C and relative humidity of 70–80% was maintained. Adults from tenth generation were used as the susceptible population (LAB strain) in this study.

RETRACTED

### 2.5. Insecticides used

Insecticide impregnated papers (0.05% Deltamethrin, 0.05% Lamdacyhalothrin, 0.75% Permethrin, 4% DDT, 0.1% Propoxur and 5% Malathion) were purchased from University Sains Malaysia and belong to four different classes of insecticides.

### 2.6. Insecticide susceptibility tests

Adult bioassay tests with six different insecticides were performed following WHO guidelines [10]. 25–30 non blood-fed adults from each population and LAB strain were exposed to insecticide impregnated papers for an hour and then shifted to retention tubes. Adult mosquitoes from the assay were maintained at laboratory condition and provided with 5% sucrose solution to feed upon. After 24 hours of insecticide exposure, mortality percentages were calculated and each experiment was run thrice. In the control, 25–30 adult mosquitoes were exposed to filter paper sprayed with acetone and carrier oil. For the calculation of knock down time (KDT) of the synthetic pyrethroids and DDT, knocked down mosquitoes were calculated after every 10 minutes during the 1 hour exposure to insecticides.

### 2.7. Synergist assay

The synergist assays were conducted using two most commonly used synergists Piperonyl butoxide (PBO)–cytochrome P_450_ (CYP_450_) inhibitor and Triphenyl phosphate (TPP)—carboxylesterases (CCEs) inhibitor. Therefore, the test was conducted in order to study the effectiveness of synergists in increasing the mortality rate of adult mosquitoes against insecticides by affecting the detoxifying enzymes. Synergists were used in their sub-lethal dose *i*.*e*., 4% PBO and 10% TPP. Thirty non-blood fed adults (from each study site and LAB strain) were exposed to synergist impregnated paper for an hour after which they were exposed to insecticide impregnated paper for an hour. The mosquitoes were then shifted to retention tube like in the adult bioassay test and mortality counted after 24 hours. The adult bioassay data was taken as positive control and exposure to insecticide-free filter paper was regarded as negative control for the synergist assay.

### 2.8. DNA extraction

Genomic DNA of 20 adult mosquitoes each from six study sites that survived after 24 hours of bioassay test against synthetic pyrethroids and DDT were extracted according to the High Salt protocol [19] with minor modifications. Individual mosquito was homogenized using digestion buffer in a 1.5 ml micro-centrifuge tube. 20 μl proteinase K was added and the samples incubated at 55–60°C in a water bath for at least 2 hours. Chloroform and sodium chloride solution was then added and the sample centrifuged at 14000 g for 15 mins. The supernatant was transferred to new micro-centrifuge tube, chilled 70% ethanol added and centrifuged at 10000 g for 5 mins. The supernatant was discarded and pellet suspended in autoclaved distilled water and stored at –20°C for further use. The same protocol was followed to extract DNA from 20 (twenty) adults of LAB strain, with no prior exposure to insecticides.

RETRACTED

### 2.9. Detection of kdr mutation

Allele-specific PCR (AS-PCR) reactions were performed using the extracted genomic DNA individually to detect two kdr mutations at the sodium channel gene, L1014F and L1014S following the standard protocol [20,21] with minor modifications. Cgd1 (5-GTGGAACTTCACCGACTTC-3), Cgd2 (5-GCAAGGCTAAGAAAAGGTTAAG-3), Cgd3 (5-CCACCGTAGTGATAGGAAATTTA-3) and Cgd4 (5-CCACCGTAGTGATAGGAAATTTT-3) primers were used to detect the L1014F mutation [20,21] and an additional primer Cgd5 (5-CCACCGTAGTGATAGGAAATTC-3) for L1014S was used in the assay. Four PCR reactions were run in parallel. Cgd1 and Cgd2 primers were combined in the first reaction, Cgd2 and Cgd3 in the second, Cgd2 and Cgd4 in third reaction and Cgd2 and Cgd5 primers combined in the fourth reaction. PCR conditions were an initial denaturation at 95°C for 15 min, followed by 30 cycles at 94°C for 45 seconds, 49°C for 45 secs, 72°C for 45 secs, and a final extension of 10 mins at 72°C. The amplified fragments were analysed on 3% agarose gels under UV light. Ethidium bromide was used to stain the agarose gel. Cgd 1–2 primers provided a product size of 540 base pair and Cgd 3, 4 and 5 primers amplified bands at 380 base pair (S1 Fig). Two PCR products amplified using Cgd1 and Cgd2 primers from each population were sequenced (Bioserve Biotechnologies (I) Pvt. Ltd.) to confirm the presence of mutations (S2 Fig).

### 2.10. Calculations

Mortality percentages against each insecticides were calculated and the mosquito populations were termed resistant (<90% mortality), susceptible (98–100% mortality) and unconfirmed resistance (90–98% mortality) accordingly [10]. In case of more than 10% mortality in control setup, the data was corrected using Abbott’s formula. Mortality percentages of adult bioassay data were subjected to one way ANOVA at 95% confidence level in SPSS software version 21.0. KDT_50_ and KDT_90_ values were also calculated using SPSS software version 21.0 at 95% confidence level by subjecting knocked down values to probit analysis.

## 3. Results

### 3.1. Mosquito collection

A total of 17,341 mosquito larvae and pupae were collected from six different sites of the two districts. Immature stages of *Anopheles sp*., Chironomids and drain flies were also found to be associated with *Cx*. *quinquefasciatus* larvae in most of the breeding habitats. Details of the mosquito collection, nature of the sampling site and its larval density, co-existence of other species are provided in Table 1.

RETRACTED

### 3.2. Adult bioassay

*Culex quinquefasciatus* adults from six different sampling sites were found to be resistant to multiple insecticides as they showed low mortality percentages against all six insecticides used in the study (Table 2). Mortality percent ranged from 7.69–36.36 for deltamethrin, 4–34.61 for lambdacyhalothrin, 11.11–36.36 for permethrin, 0–34.61 for DDT, 0–18.18 for propoxur and 0–8 for malathion (Table 2). KDT_50_ and KDT_90_ values against synthetic pyrethroids and DDT ranged from 157.04–1132.28 minutes (Table 3). Such high KDT values show a greater amount of time taken by the insecticides to knockdown 50% and 90% mosquito population thereby leading to the onset of resistance.

**Table 2:** Mortality rate (in percent) of *Cx*. *quinquefasciatus* from Coochbehar and Malda districts against six insecticides. M%- mortality percentage; S.E- Standard error; n-total number of mosquito adults.

Sampling site	Deltamethrin M% ± S.E	Lambdacyhalothrin M% ± S.E	Permethrin M% ± S.E	DDT M% ± S.E	Propoxur M% ± S.E	Malathion M% ± S.E
COB	8.00 ± 0.62 (n = 90)	11.11 ±0.64 (n = 84)	23.08 ±0.10 (n = 78)	4.00 ±0.09 (n = 86)	18.18 ±0.13 (n = 90)	3.70 ±0.28 (n = 82)
TFG	36.36 ±0.37 (n = 87)	34.61 ±0.40 (n = 79)	36.36 ±1.83 (n = 90)	34.61 ±0.41 (n = 78)	10.00 ±0.09 (n = 90)	0.00 ±0.00(n = 79)
MEK	7.69 ±0.15 (n = 85)	9.67 ±0.90 (n = 90)	31.03 ±0.81 (n = 84)	6.25 ±0.12 (n = 76)	3.57 ±0.17 (n = 81)	3.22 ±0.56 (n = 78)
MLT	12.00 ±0.61 (n = 90)	4.00 ±0.13 (n = 86)	11.11 ±0.64 (n = 82)	0.00 ±0.00 (n = 82)	3.45 ±0.28 (n = 83)	8.00 ±0.41 (n = 90)
SAM	11.54 ±1.85 (n = 90)	7.32 ±0.67 (n = 78)	14.28 ±0.37 (n = 89)	3.57 ±0.10 (n = 84)	0.00 ±0.00 (n = 89)	0.00 ±0.00 (n = 85)
HCP	14.28 ±0.73 (n = 87)	34.61 ±1.28 (n = 90)	20 .00±0.52 (n = 78)	0.00 ±0.00 (n = 90)	12.90 ±0.16 (n = 81)	0.00 ±0.00 (n = 83)
LAB strain	100 ± 0.00 (n = 90)	99.36 ± 0.26 (n = 90)	100 ± 0.00 (n = 90)	98.92 ± 0.09 (n = 90)	100 ± 0.00 (n = 90)	100 ± 0.00 (n = 90)

**Table 3:** KDT_50_ and KDT_90_ values (in minute) of *Cx*. *quinquefasciatus* populations against Synthetic pyrethroids and DDT.

Sampling site	Deltamethrin		Lambdacyhalothrin		Permethrin		DDT	
	KDT_50_	KDT_90_	KDT_50_	KDT_90_	KDT_50_	KDT_90_	KDT_50_	KDT_90_
COB	189.38	382.77	199.48	412.43	221.19	478.14	378.90	1132.28
TFG	199.80	494.27	378.90	1132.28	212.91	614.45	378.89	1132.28
MEK	378.90	1132.28	157.04	315.68	129.57	246.38	221.19	478.14
MLT	344.56	984.90	344.50	984.87	171.30	331.14	------	------
SAM	130.05	238.83	391.12	1055.05	143.17	273.04	248.85	752.60
HCP	141.01	269.26	116.31	208.73	103.53	179.80	------	------
LAB strain	42.30	83.56	55.62	107.28	58.17	96.24	49.25	103.24

RETRACTED

### 3.3. Synergist assay

Result of the synergist assays showed a non-significant increase in the mortality rate of *Cx*. *quinquefasciatus* adults against insecticides used (Table 4). Susceptibility of *Cx*. *quinquefasciatus* populations to synthetic pyrethroids and DDT could not be restored with the use of two synergists though there was an increase in the mortality rate. Likewise, mortality percentage against malathion and propoxur showed an increase when compared to the mortality rate of adult bioassay test but the observed resistant status could not be reverted to susceptible indicating only a minor involvement of major detoxifying enzymes behind resistance in the two districts. Thus, CYP_450_s and CCEs are probably not the major mechanism of resistance in the populations under study.

**Table 4:** Mortality rate (in percent) of *Cx*. *quinquefasciatus* populations after exposure to synergists and insecticides.

Sampling site	Synergist	Deltamethrin M% ± S.E	Lambdacyhalothrin M% ± S.E	Permethrin M% ± S.E	DDT M% ± S.E	Propoxur M% ± S.E	Malathion M% ± S.E
COB	PBO	30.43±0.82	29.24±0.58	32.81±0.05	7.73±0.04	31.03±0.21	20.80±0.34
TFG		9.09±0.06	35.00±1.63	75.00±0.72	5.56±0.17	23.08±0.57	3.20±0.03
MEK		93.10±1.92	51.35±2.84	9.00±0.19	87.50±0.06	78.79±0.76	85.18±0.45
MLT		23.85±0.18	16.22±0.67	21.36±0.42	7.54±0.76	14.81±0.07	14.81±1.29
SAM		21.43±0.36	12.00±0.94	19.23±0.42	9.57±0.05	15.21±0.43	10.71±0.08
HCP		88.46±0.54	68.75±0.68	61.90±0.61	20.00±0.16	48.39±0.63	21.30±0.17
LAB strain		100±0.00	100±0.00	100±0.00	99.54±0.42	100±0.00	100±0.00
COB	TPP	22.83±0.28	35.31±1.57	27.73±0.18	6.91±0.06	29.42±0.82	21.74±0.43
TFG		15.00±0.16	85.71±0.09	70.37±0.49	25.00±0.18	5.26±0.46	11.11±0.08
MEK		87.50±0.54	86.21±0.43	60.00±1.57	84.85±1.59	79.17±1.81	83.33±2.57
MLT		10.34±1.37	15.00±0.04	4.76±0.83	12.50±0.48	10.71±0.75	13.04±0.46
SAM		15.79±0.08	12.12±0.81	24.24±0.07	6.91±0.08	17.24±0.31	18.37±0.32
HCP		77.5±0.25	73.91±0.24	30.77±1.23	4.00±0.03	3.33±0.06	11.29±1.90
LAB strain		100±0.00	100±0.00	100±0.00	100±0.00	100±0.00	100±0.00

### 3.4. Detection of kdr

The PCR analysis of kdr allele showed presence of 5 genotype frequencies in varying number in all study areas. L1014F mutation was found to occur in all study sites with maximum resistant homozygote (F/F) genotype frequency in Malda (30%) followed by MEK (25%) and HCP (25%) (Table 5). TFG showed highest heterozygote genotype frequency (L/F) of 35% followed by COB (25%). The homozygote wild genotype frequency (L/L) was comparatively higher ranging from 35–50%. The mosquito population under study showed an average resistant allele frequency (F) to be at 28.75% of the entire population with Malda showing the highest allele frequency *i*.*e*., 37.5% of the population. No kdr mutation was observed in LAB strain (susceptible population).

RETRACTED

**Table 5:** Genotypic and allelic frequencies of L1014F and L1014S kdr mutations in *Culex quinquefasciatus* from two districts of West Bengal.

Sampling site	Genotype frequency (%)					Allele frequency			F_IS_
	LL	LF	FF	LS	SS	L	F	S	
COB	50	25	10	10	5	0.675	0.225	0.1	-0.447
TFG	35	35	0	30	0	0.675	0.175	0.15	-1.646
MEK	40	15	25	10	10	0.525	0.325	0.15	0.161
MLT	35	15	30	10	10	0.475	0.375	0.15	0.182
SAM	40	20	20	15	5	0.575	0.3	0.125	-0.242
HCP	40	15	25	10	10	0.525	0.325	0.15	0.161

No FS individuals were found so it has been omitted from the table. F_IS_ is Wright Index of inbreeding coefficient which measures the probability of inbreeding in a population due to non-random mating. When F_IS_ is a negative value the population is an outbreed population; F_IS_ < 0.3 indicates within range inbreeding. Bold value indicates inbreed population.

PCR analysis of L1014S mutation in the voltage-gated sodium channel gene also showed the presence of mutation but to a lower extent when compared to L1014F mutation in the same population (Table 5). Highest heterozygote genotype frequency (L/S) was shown by TFG (30%) and homozygote mutated genotype frequency (S/S) ranged from 5–10% in all of the populations under study. COB and TFG populations showed highest wild allele frequency (L) (67.5%), SAM 57.5% and the rest three populations showed 47.5–52.5% allele frequency (Table 5). Resistant allele frequency ranged from 10–15%.

## 4. Discussion

The prime objective of the present study was to assess the insecticide susceptibility status of *Cx*. *quinquefasciatus*, a vector of lymphatic filariasis in two filariasis endemic districts of northern West Bengal against four classes of insecticides and also to find out the presence of kdr mutation in the vector population and its association with resistance to synthetic pyrethroids and DDT. High larval density observed in both the districts can be attributed to the ample habitat provided for mosquito breeding along with little or no control measures taken against this vector of lymphatic filariasis.

The field mosquito population showed severe resistance to propoxur—a carbamate insecticide (Table 2). The World Health Organisation Pesticide Evaluation Scheme (WHOPES) recommends 2 hours of exposure period to propoxur for *Cx*. *quinquefasciatus*. However, in this study to maintain the homogenity of the experiment, 1 hour exposure time was followed for all six insecticides. Till date, there is no report on propoxur being used as a mosquitocide in India [9] thereby indicating the indirect exposure of *Cx*. *quinquefasciatus* to other insect repellents that contain propoxur and are used in the household. The indoor resting habit of this vector might have added upon its exposure to such repellents. Similar findings on resistance of *Cx*. *quinquefasciatus* to carbamate insecticides have been reported by researchers [10,22]. Likewise, the adult bioassay test of field caught population of *Cx*. *quinquefasciatus* showed severe resistance to malathion with three (TFG, SAM, HCP) out of six population showing zero mortality and MLT with highest mortality rate of 8%. Malathion belonging to organophosphate class of insecticide is not directly applied against mosquito as a part of mosquito control programmes but applied on large scale in the agricultural sector. Therefore, severe resistance to malathion observed in the present study may be linked to the indirect exposure of the vector population to malathion residues from the agricultural run-off which accumulate in the nearby drains and channels that might harbor *Cx*. *quinquefasciatus* populations. The two districts under study–Coochbehar and Malda depends largely on the agricultural practices, Coochbehar cultivating mainly paddy, tobacco and jute and the district of Malda being dependent on prime orchard crops like mango, banana and litchi for their economy. Thus, the contamination of *Cx*. *quinquefasciatus* breeding habitats by the seeping of excessive malathion used in the agricultural practices in the adjoining drains leads to indirect exposure of *Cx*. *quinquefasciatus* to the insecticide thereby bringing about the onset of resistance development in the vector population [23,24].

RETRACTED

Resistance to malathion in *Cx*. *quinquefasciatus* has been reported to be associated with an increase in the production of non specific esterases [10,25,26] and that of carbamate by an increased level of CCEs activity primarily and rarely by CYP_450_s and GSTs activity [27]. No significant increase in mortality percent of *Cx*. *quinquefasciatus* in the synergism test with TPP except for MEK population show that the CCEs were not the major mechanism of resistance development in the studied populations of mosquito vector of Coochbehar and Malda districts. Moreover, similar result on the use of PBO suggest little involvement of CYP_450_s in resistance development as well thereupon providing a hint on the presence of other mechanisms of resistance mainly target-site mutation behind the observed resistance to malathion and propoxur. Organophosphates and carbamate being acetylcholinesterase inhibitor insecticides target the ace-1 gene [12]. Further studies on unveiling the molecular mechanism behind resistance development against these two classes of insecticides should be an important focus and carried out by mapping the presence of mutation in ace-1 gene which in turn leads to inhibition on the proper functioning of acetylcholinesterases.

Low mortality rates in the studied mosquito populations against three synthetic pyrethroids (deltamethrin, lambdacyhalothrin, permethrin) suggest a severe degree of resistance level against this insecticide class. This observed resistance in *Cx*. *quinquefasciatus* populations of two filariasis endemic districts of West Bengal is of immense concern owing to the fact that synthetic pyrethroids are the only class of insecticides that are used in the insecticide impregnated bed nets as a control program against malaria as recommended by WHO in West Bengal and around the globe [28] and for indoor spraying against mosquitoes owing to their rapid action and safety to humans. Many studies have already reported on the inefficiency of pyrethroid treated bed nets to counter *Cx*. *quinquefasciatus* and malarial vector *Anopheles* species [29,30]. Though there are no reports on the application of pyrethroid insecticides directly on *Cx*. *quinquefasciatus* in West Bengal, the domestic use of synthetic pyrethroids to control household pests and combat the nuisance caused by mosquito biting may be considered as the most probable cause of resistance development to synthetic pyrethroids in *Cx*. *quinquefasciatus* as observed in the current study. Synthetic pyrethroids-containing products like mosquito coils, repellent oils, fumigants and sprays add upon the resistance development of *Cx*. *quinquefasciatus* to synthetic pyrethroids as this vector being anthropophilic [31] and the adults rest indoors along with *Aedes* mosquitoes, come into direct contact to the insecticide class. Moreover, the application of pyrethroids in agricultural practices in Coochbehar and Malda districts together with organophosphates may create insecticide selection pressure on the vector population. This secondary resistance in non-target mosquito population has also been reported in a previous study from sub-Himalayan West Bengal [32]. Similarly, resistance observed against DDT might also be linked to the secondary exposure of widespread use of DDT in the vector management programs [33]. The two districts apart from being endemic to filariaisis are also endemic to dengue thereby increasing the probability of untargeted exposure to insecticides aimed at controlling the *Aedes* mosquito populations but applied mostly on drains- the natural habitat of *Culex* mosquitoes.

RETRACTED

The higher KDT_50_ and KDT_90_ values in the study (Table 3) show a slower effect of synthetic pyrethroids and DDT on *Cx*. *quinquefasciatus* from all six studied sites. As pyrethroids are mainly known for their rapid knock down effect on the target, longer knock down time taken by the vector population depicts an alternation in their target site thereupon imparting a negative impact on the insecticide receptor binding in the mosquito vector [34]. This observation is well supported by the results of synergist assay test where both PBO and TPP exposure prior to DDT and pyrethroids exposure did not have a significant increase in mortality rate and was unable to revert the resistance status of *Cx*. *quinquefasciatus* (Table 4). PBO and TPP are chemical synergists which when combined with insecticides inhibit the major detoxifying enzymes of vector thereby rendering the vector population susceptible to insecticides. Resistance to synthetic pyrethroids in insects is caused by an increased quantitative level of CYP_450_s metabolic enzymes [35,36] while synergist PBO inhibit the same [37] therefore suggesting major role of other mechanisms of resistance apart from the metabolic enzymes in *Cx*. *quinquefasciatus* from two districts of West Bengal. Skovmand *et al*., 2018 [38] also reported similar indifference in mortality percentage of *Cx*. *quinquefasciatus* against pyrethroids with the use of PBO though there are studies that contrast such findings [39,40]. The practice of incorporating PBO into pyrethroid-treated long lasting insecticide impregnated bed nets (LLINs) [37] may therefore yield below expected results in controlling the vector population in these two districts.

ASPCR analysis of L1041F mutation in the *Cx*. *quinquefasciatus* population in the two districts of West Bengal showed that the homozygote resistant genotype frequency ranged from 0–30%. In MLT 30% of the tested mosquito population was found to have the dominant resistant genotype frequency. HCP in the same district and MEK in Coochbehar district showed 25% resistant genotype frequency. This finding of the present study is of prime concern due to the high numbers of resistant homozygote in the population. Though kdr mutation is a recessive trait with dominant phenotype arising only in the presence of two homozygote mutant alleles yet, COB, TFG and SAM should also not be neglected because of their low homozygote resistant genotype frequency as these populations show high heterozygote genotype frequency (L/F). Moreover, low susceptible wild genotype frequency may cause problem in the long run of vector management with chemical insecticides as in high intensity of insecticide selection pressure, the lack of susceptible mosquitoes to pass their genes to the next generation may lead to irreversible state of insecticide resistance [13].

RETRACTED

Mutation in the 1014 codon of voltage-gated sodium channel gene from leucine to phenylalanine is the most common and widely studied kdr mutation in insects though L1014S (leucine to serine), L1014C (leucine to cysteine) and L1014H (leucine to histidine) mutations have also been reported [41]. Presence of L1014F mutation in *Cx*. *quinquefasciatus* have been studied and reported from sub-Himalayan West Bengal in a previous study [42], India [21] and from different regions of the world [11,13,20,39,43,44]. However, L1014S mutation in the voltage-gated sodium channel gene in *Cx*. *quinquefasciatus* was not reported earlier. Higher survival rate of the studied mosquito population against synthetic pyrethroids and DDT together with the ineffectiveness of synergists to restore the susceptibility status of mosquito population and high frequency of L1014F mutation observed in the study indicates the association of kdr mutation with insecticide resistance in *Cx*. *quinquefasciatus* from six study sites of two filariaisis endemic districts. Moreover, there are similar findings of correlation between kdr mutation and inefficiency of the insecticides to control the vector population [45–47]. On the contrary, few studies differ from the above findings where mosquito vectors with high kdr frequency still show high mortality when treated with pyrethroid insecticides [48,49]. Thus, kdr mutation at DNA level alone is not sufficient to produce a resistant phenotype unless combined with RNA transcription [50].

Comparatively higher survival rate of *Cx*. *quinquefasciatus* to DDT than synthetic pyrethroids might be linked to the presence of L1014S mutation in the present study as this mutation is said to confer higher resistance to DDT than to pyrethroids [11,20,47]. However, the presence of L1014S mutation in the study in low frequency when compared to L1014F mutation suggest the role of detoxifying enzymes apart from kdr mutation in the development of resistance against DDT in the mosquito population [11,35]. The phenomenon of cross resistance between DDT and synthetic pyrethroids can also not be ruled out due to the high frequency of L1014F mutation in the studied population [39]. Though, different insecticide selection pressure combined with environmental factors influence the presence of a particular type of kdr mutation in the vector population [34], secondary mutations occurring at the cytoplasmic portion of sodium channel further increase the resistance level associated with mutation at 1014 codon [51].

RETRACTED

## 5. Conclusion

This study first reports resistance status of wild *Cx*. *quinquefasciatus* populations to commonly used insecticides from filariasis endemic districts of northern West Bengal and also the presence of two kdr mutations pertaining to the observed resistance. To our knowledge this is the first report of the presence of L1014S mutation in *Cx*. *quinquefasciatus*. Prior to this study, L1014S mutation was reported from *Cx*. *pallens* and *Cx*. *pipiens* only. The observed resistance can be linked to the presence of kdr mutations L1014F and L1014S in the sodium channel gene. Involvement of metabolic resistance in the studied populations was not found in the present study. Though, the presence of kdr mutation indicates resistance status in vectors other mechanisms of resistance and several co-factors combinely work to impact upon insecticide resistance level. Resistance development at a particular site depends on insect biology, dominant mechanisms of resistance and history on previous strategies taken to control vector population. As such, studying and monitoring the site-specific resistance intensity along with the mechanisms associated is important. Transmission of vector-borne diseases will increase in the years ahead especially those carried by *Culex* mosquitoes due to their opportunistic behavior, adaption to climate changes and poor sanitary conditions [52] thereby further indicating on the need of mapping insecticide resistance of wild mosquito populations from different sub-regions of tropical and sub-tropical countries.

## Supporting information

S1 Fig Gel electrophoresis image showing different bands obtained through allele-specific PCR (AS-PCR) of kdr mutation in voltage-gated sodium channel gene in *Culex quinquefasciatus* from West Bengal. L1 and L7: 100–1500 bp DNA ladder, L2: PCR product at 540 bp depicting the region of mutation, L3, L4 and L5: PCR product at 380 bp depicting L1014F, L1014L and L1014S alleles respectively, L6: negative control.
(TIF)

S2 Fig Chromatogram obtained from sequencing of PCR product. a. Wild type with no mutation in 311^th^ or 312^th^ Position (Leucine), b. Mutation from A to T in 312^th^ Position (Leucine to Phenylalanine), c. Mutation from T to C in 311^th^ Position (Leucine to Serine). Mutated base has been marked with an arrow.
(TIF)
